# Positive Effects against UV-A Induced Damage and Oxidative Stress on an* In Vitro* Cell Model Using a Hyaluronic Acid Based Formulation Containing Amino Acids, Vitamins, and Minerals

**DOI:** 10.1155/2018/8481243

**Published:** 2018-06-26

**Authors:** Antonietta Stellavato, Anna Virginia Adriana Pirozzi, Stella Donato, Ilaria Scognamiglio, Sabrina Reale, Alba Di Pardo, Stefania Filosa, Valentina Vassallo, Gilberto Bellia, Mario De Rosa, Chiara Schiraldi

**Affiliations:** ^1^Università della Campania Luigi Vanvitelli (ex Second University of Naples), Department of Experimental Medicine, Section of Biotechnology, Medical Histology and Molecular Biology, Via Luigi De Crecchio No. 7, 80138 Naples, Italy; ^2^Institute of Biosciences and BioResources-CNR, UOS Naples, Italy; ^3^IRCCS Neuromed, Pozzilli, Italy; ^4^IBSA Farmaceutici Italia Srl, Lodi, Italy

## Abstract

Ultraviolet (UV) radiations are responsible for skin photoaging inducing alteration of the molecular and cellular pathways resulting in dryness and reduction of skin elasticity. In this study, we investigated,* in vitro*, the antiaging and antioxidant effects of hyaluronan formulations based hydrogel. Skinkò E, an intradermic formulation composed of hyaluronic acid (HA), minerals, amino acids, and vitamins, was compared with the sole HA of the same size. For this purpose, HaCaT cells were subjected to UV-A radiations and H_2_O_2_ exposure and then treated with growth medium (CTR) combined with M-HA or Skinkò E to evaluate their protective ability against stressful conditions. Cells reparation was evaluated using a scratch* in vitro* model and Time-Lapse Video Microscopy. A significant protective effect for Skinkò E was shown with respect to M-HA. In addition, Skinkò E increased cell reparation. Therefore, NF-kB, SOD-2, and HO-1 were significantly reduced at the transcriptional and protein level. Interestingly, *γ*-H2AX and protein damage assay confirmed the protection by hyaluronans tested against oxidative stress. G6pdΔ ES cell line, highly susceptible to oxidative stress, was used as a further cellular model to assess the antioxidant effect of Skinkò E. Western blotting analyses showed that the treatment with this new formulation exerts marked antioxidant action in cells exposed to UV-A and H_2_O_2_. Thus, the protective and reparative properties of Skinkò E make it an interesting tool to treat skin aging.

## 1. Introduction

Dermal exposure to UV is responsible for skin photoaging [1]. Ultraviolet A (UV-A) represents 90% of all UV radiations [2]. However, UV-B and UV-A may challenge epidermal cells (keratinocytes, melanocytes, Langerhans', and Merkel's cells) possibly impairing the metabolism of these cells [3]. Besides, UV-A photons tend to damage the skin even after a short exposure [4], inducing the phosphorylation of JNK through an increase of intracellular ROS in human keratinocytes (HaCaT) [5]. Other manuscripts reported the impact of ROS on keratinocytes, proving also in this cell model the specific external stress, which can generate oxygen species in the cells [6]. Also, extensive UV-A exposure to DNA damage similar to UV-B exposure is reported by Mouret and collaborators [7]. These radiations penetrated into the deep area of the dermis and destroyed the connective collagen and elastin fibres in the tissue, challenging the cellular homeostasis. As a result, the macromolecular assembly of collagen and elastin in the skin may be impaired or modified, thus causing the skin to become thinner and lose elasticity [8]. The process leads to the catabolism of extracellular matrix components (collagens and proteoglycans) with a loss of matrix [9]. This phenomenon is particularly due to matrix metalloproteinases expression. A strong degradation of type I collagen also occurs in irradiated skin compared with nonirradiated skin [10]. In addition, excessive exposure induces alteration of the biomechanical properties of dermal connective tissue resulting in dryness and reduced skin elasticity [11]. These changes are coupled with DNA damage induced by reactive-oxygen species (ROS) production [12] that not only lead to premature aging of the skin but also increase the risk of contracting skin cancer. Moreover, ROS, inducing apoptosis, reduces the number of skin fibroblasts and decreases their regenerative capacity, leading to increased skin sagging [13]. Furthermore, environmental pollutants may contribute to prompt symptoms of extrinsic skin aging, including coarse wrinkles, irregular pigment spots, and elastosis [14]. Thus, the identification of new compounds, which are effective in protecting skin cells, is an important tool to prevent and/or to contrast the damage induced by ultraviolet radiation. Currently, there is a great tendency to use different skin care product formulations, considering their effect on the reduction of free radicals production generated from ultraviolet radiation. To date, stimulation of skin biorejuvenation is facilitated by minimally invasive intradermal injections of biologically active substances [15, 16] such as hyaluronic acid- (HA-) based gels and dermal fillers [17] alone or in combination with other molecules [18, 19]. Reports show that HA accelerates* in vitro* processes related to wound healing [20] and* in vivo* tissue regeneration, increasing the production of extracellular matrix components [21] that reduce the signs of aging [22]. In particular, HA enhances hydration in the extracellular space due to its ability to attract water molecules [23] and induces optimal physiological conditions in the extracellular matrix for cell proliferation [24] and the organization of fibroblasts. Recently, the protective effect of HA has been proposed as an effective tool against skin damage [25]. An intradermic formulation containing linear HA and antioxidants, which is able to suppress oxidative stress-induced apoptosis in skin fibroblasts, can be a potential treatment for maintaining healthy youthful skin. In the present study, we evaluated the hydrodynamic and biological characterization of a compound containing linear HA plus a mixture of vitamins, antioxidants, and minerals named VISCODERM™ Skinkò E [14]. The aim of this work was to understand the mechanism of the action of medium molecular weight HA (M-HA) and the same HA added with vitamins, antioxidants, and minerals on* in vitro* models of oxidative damage.

## 2. Materials and Methods

### 2.1. Materials

The M-HA was obtained in our laboratory by heterogeneous hydrolysis acid of HA 1200 kDa pharma grade, kindly provided by Altergon s.r.l., following the procedure reported in D'Agostino and collaborators (2017) [25]. In particular, size-exclusion chromatography, equipped with a triple detector, permitted the following characterization: 500±80 kDa, Mw/Mn=1,6. Intrinsic Viscosity=1,1±0,2 m3/kg [25]. The compound was then dissolved in phosphate-buffered saline (PBS) (6,4 mg/ml in PBS) and microfiltered (0,22 *μ*m) in order to be sterilized. Endotoxin content was lower than 0,05 EU/mg. Skinkò E (6,4 mg/mL) was kindly provided by IBSA Farmaceutici Lodi-Italia. This intradermic formulation was released by dissolving HA raw material with an intrinsic viscosity ranging from 0,90 to 1,34 m3/kg. Composition for 5 mL vial, as reported in the commercial leaflet contains, apart from the linear M-HA, biotechnological origin. Buffered preservation media contain (1) inorganic salts: Ammonium molybdate, ammonium metavanadate, calcium chloride, iron sulfate, potassium chloride, copper sulfate, magnesium chloride, manganese sulfate, sodium acetate, sodium hydrogen carbonate, sodium chloride, sodium hydrogen phosphate, sodium metasilicate, sodium selenite, tin chloride, and zinc sulfate; amino acids: alanine, arginine, asparagine, aspartic acid, cysteine, glutamine, glutamic acid, glycine, histidine, isoleucine, leucine, lysine, methionine, phenylalanine, proline, serine, threonine, tryptophan, tyrosine, valine, and adenine; vitamins: biotin (vitamin H), calcium pantothenate (vitamin B5), choline chloride, folic acid (vitamin B9), inositol, nicotinamide, pyridoxine (vitamin B6), riboflavin (vitamin B2), thiamine (vitamin B1), cyanocobalamin (vitamin B12); antioxidants: lipoic acid; others: inositol, glucose, putrescine, and sodium pyruvate. MHA and Skinkò E were opportunely diluted 1:1 with complete growth medium, supplemented with fetal bovine serum (FBS) to obtain 1% v/v FBS for the time-lapse experiment. For all experiments, Skinkò E and M-HA solutions were diluted 1:2 from stock solutions of 0,64% w/w in cell medium and then used at a 0,32% v/v final concentration.

### 2.2. Cell Culture

The immortalized human keratinocyte cell line (HaCaT) was obtained from Istituto Zooprofilattico, (Brescia, Italy). Cells were maintained at 37°C in a humidified atmosphere containing CO_2_ (5% v/v) in Dulbecco's modified Eagle's medium supplemented with 10% fetal bovine serum, 2 mM glutamine, and 1% penicillin/streptomycin. For the experiments, HaCaT cells were incubated with freshly prepared dilutions of the M-HA 0,32% w/v and Skinkò E 0,32% w/v, and in growth medium, for the specified time and concentration range.

A mouse embryonic stem (ES) cell line, which was engineered through the deletion of the glucose-6-phosphate-dehydrogenase gene (G6pdΔ cells) [26] and the wild type (WT) ES cell, was maintained in an undifferentiated state by culture on a monolayer of mitomycin C inactivated fibroblasts, in the presence of leukemia-inhibiting factor (LIF) [27]. Cells were seeded, at equal density on gelatin-coated plates, 48 hours before treatment. Cells were treated with 100 mU/ml (WT ES) or 10 mU/ml mU (G6pdΔ ES) of glucose oxidase (GOX; Sigma-Aldrich) for 30 minutes and then incubated in the presence of M-HA or Skinkò E and harvested after 8 hours.

### 2.3. Sample Preparation

VISCODERM® Skinkò E formulation was concentrated on a polyethylene sulfate membrane with a nominal molecular weight limit (NMWL) of 3 kDa (Amicon Ultra 0.5 mL Centrifugal filter: Ultracel 3 kDa, Millipore). The concentration was diafiltered using 2 volumes of HPW (High Purified Water). Successively, the ultrafiltration (UF) retentate on the 3 kDa centricon tube was recovered and eventually diluted for the hydrodynamic characterization by SEC-TDA; whereas, the permeate 3 kDa was analyzed by uronic acid assay (E.P. ed 5.0: 2.2.25). This last assay quantified the residual HA in the permeate and diafiltered sample that accounted for about the 25% w/w of the initial HA amount. Therefore, the permeate 3 kDa contained all the Skinkò E components and a residual 1,84 mg/mL of HA. This was diluted 1:2, tested as for Skinkò E, and thus, the final concentration of HA in the cell's plate was 3,2 mg/mL for the complete formulation and only 0,92 mg/mL for the permeation. In this case, the HA effect should be reduced with respect to the other compounds present in the formulation.

### 2.4. Hydrodynamic Characterization SEC-TDA

The chromatographic analyses of ultra-filtered retentate Skinkò E and M-HA using size-exclusion chromatography coupled with triple detection array (SEC-TDA by Viscotek Malvern Instruments, UK) were performed. The details of the system and the analytical conditions have been reported by La Gatta et al. (2010) [28]. The molecular size, molecular weight distribution, polydispersity, and the intrinsic viscosity of the samples have been derived for a complete hydrodynamic characterization.

### 2.5. Wound Healing In Vitro Model on HaCaT

The* in vitro* scratch assay procedure has been fully previously described [18, 20]. In brief, 12 wells (precoated with collagen) were seeded with HaCaT (1,5×10^3^cells/cm^2^) and incubated for 48 hours until complete confluence was reached, in order to test the effect of M-HA and Skinkò E (0,32% w/v), respectively, on the rate of wound closure, monitored by Time-Lapse Videomicroscopy (TLVM). Fresh serum-supplemented medium with 1% v/v FBS was used as a control. The images of the scratched monolayers were captured every 60 minutes and analyzed using OKO Vision 4.3 software (Okolab, Italy) [25].

### 2.6. Analysis of SOD-2 and HO-1 through qRT-PCR

To test* in vitro* antioxidant activity, HaCaT cells were treated with M-HA and Skinkò E for 4 hours, with and without preexposure to U-VA radiation (*λ*_max_ 365 nm) for 4 minutes [29]. For the analysis of gene expression, total RNA was extracted, using Trizol, according to the manufacturer's procedures (Invitrogen, Milan, Italy). Retrotranscription was performed using Reverse Transcription System Kit (Promega, Milan, Italy). PCR was then performed using iQ™ SYBR1-Green Supermix (Bio-Rad Laboratories s.r.l., Milan, Italy) to analyze the expression levels of superoxide dismutase-2 (SOD-2), heme oxygenase 1 (HO-1), and hypoxanthine guanine phosphoribosyl transferase (HPRT), using the specific primer pairs designed with Beacon Designer software (Bio-Rad Laboratories s.r.l., Milan, Italy). Primer sequences have been reported in Table 1 and the amplification conditions have been fully described in Stellavato and collaborators (2016) [30]. All PCR reactions were performed in triplicate and the relative expression of specific mRNA with respect to the hypoxanthine guanine phosphoribosyl transferase (HPRT) housekeeping gene. The comparative threshold method 2^−ΔΔCt^ (ΔΔCt = difference of ΔCt between HA treated cells and control) has been used to calculate the fold-change of genes and the results have been expressed as normalized fold expression, compared with controls using the Bio-Rad iQ™5 software (Bio-Rad Laboratories s.r.l.).

### 2.7. Western Blotting for NF-kB and HO-1 as Inflammatory Markers

For the evaluation of western blotting, HaCaT cells were treated with M-HA and Skinkò E for 24 h with and without preexposure to U-VA radiation (*λ*_max_ 365 nm) for 4 minutes [29]. The proteins were extracted using a RIPA lysis buffer and the concentrations were determined using the Bio-Rad protein assay reagent (Bio-Rad Laboratories, Milan Italy). Equal amounts of proteins (30 *μ*g) were loaded on a SDS-PAGE and transferred them to a nitrocellulose membrane [31]. The filters were incubated with antibodies against the nuclear factor kappa-light-chain-enhancer of activated B cells (NF-kB; rabbit polyclonal IgG C-20; 1:200 v/v ), heme oxygenase 1 (HO-1; goat polyclonal IgG C-18; 1:200 v/v), and actin (actin; goat polyclonal IgG I-19; 1:500) at room temperature for 2 hours. Membranes were washed three times for 10 minutes and incubated with a 1:5000 dilution of horseradish peroxidase-conjugated anti-rabbit antibodies and with a 1:10000 dilution of horseradish peroxidase-conjugated anti-goat antibodies for 1 hour, respectively. All antibodies are purchased from Santa Cruz Biotechnology, CA, USA. Blots were developed using the ECL system according to the manufacturer's protocols (Amersham Biosciences). Extracted proteins from Skinkò E treated WT and G6pdΔ ES cells [32] and untreated cells were analyzed using PARP antibody (New England Biolabs.). Actin antibody was used as the gel loading control. The same procedure of western blotting was followed to analyze *γ*-H2AX (primary antibody anti-*γ*H2AX: Cat No. 05-636 from Millipore, MA, USA) as specific biomarker of DNA damage prompted by oxidative stress.

### 2.8. Antioxidant In Vitro Activity Using T-Bars Assay on HaCaT

Reactive aldehydes were assessed by measuring thiobarbituric acid-reactive substances (TBARS), as described previously [32]. The effect of Skinkò E on HaCaT cells (2,0 x10^5^) was tested in four different experimental setups:

1. To test the effect on the poststress process, the cells were pretreated for 30 minutes with 50 *μ*M H_2_O_2_ and then incubated with M-HA and Skinkò E (0,32% v/v) for 24 hours.
2. To test the antioxidant activity, M-HA and Skinkò E were applied simultaneously with 50 *μ*M H_2_O_2_ (30 min) or exposed to a U-VA radiation (*λ*_max_ 365 nm) for 4 minutes.
3. To test the effect of the permeate (3 kDa) Skinkò E formulation, with respect to complete Skinkò E formulation on HaCaT cells, the cells were pretreated with 50 *μ*M H_2_O_2_ or exposed to a U-VA radiation (*λ*_max_ 365 nm).

The protein concentrations were determined using the Bio-Rad protein assay reagent (Bio-Rad Laboratories, Milan Italy). A TBARs assay (thiobarbituric acid-reactive substances) was performed on aliquots of membranes which were extracted (10 *μ*l) and added to 2 ml of TBA-TCA (TCA 15% w/v, TBA 0,3% w/v in HCl 0,12 N) solution at 100°C for 30 minutes. The chromogen, produced by the stoichiometric reaction of aldehydes (malondialdehyde (MDA)) with thiobarbituric acid (TBA), was quantified by spectrophotometric reading at a wavelength of 532 nm. The amount of TBARs was expressed as a percentage of lipid peroxidation and then normalized with respect to the control.

## 3. Results

### 3.1. Molecular Weight, Polydispersity, and Intrinsic Viscosity Determination by SEC-TDA

The Skinkò E product (Viscoderm Skinkò E VEVU04), analyzed by SEC-TDA, contains HA with an intrinsic viscosity of 0,97±0,2 m^3^/kg, which is within the expected range (as reported by the producer). A comparative analysis of Skinkò E and M-HA (produced by our laboratory) showed similarities to the chromatographic profile (see Figures 1(a)-1(b)) and derived analytical software parameters. Detailed analyses of molecular distribution highlighted a molecular weight fraction above 700 kDa of 14%, whereas over 40% resulted above 400 kDa for both Skinkò E and M-HA. These results confirmed comparable molecular weight distributions between samples, thus permitting a correct biological/cellular comparison between the treatments.

### 3.2. In vitro Scratch Assay Using Time-Lapse Video Microscopy (TVLM)

Wound healing experiments showed that the scratch closure occurred at a faster rate in the presence of Skinkò E and M-HA (the control cells being in normal medium). Between the two M-HA based samples analysed, the Skinkò E acted faster than M-HA. In particular, in wound closure, the sole M-HA achieved 70% of reparation at 14 hours compared with 18 hours for the control. Surprisingly, a higher performance was found for Skinkò E. In fact, samples treated with Skinkò E reached the same repair target (70%) within 9 hours (see Figure 2), corresponding to a 2-fold increase of the reparation rate with respect to the control and also a significant 30% improvement with respect to the sole M-HA.

### 3.3. Gene and Protein Expression Analyses

M-HA and Skinkò E showed the capability of preventing UV-A stress,* in vitro,* in experiments accomplished using a model recently described by Almeida and collaborators (2015) [25]. SOD-2 and HO-1 were markedly reduced at the transcriptional level. In particular, SOD-2 and HO-1 gene expression, as reported in Figure 3, were significantly downregulated with respect to UV-A treatment in the presence of Skinkò E. SOD-2 was reduced 2,4-fold, and HO-1 2-fold, with respect to M-HA alone. Similarly, the protein levels of NF-kB and HO-1 (see Figures 4(a)-4(b)) significantly decreased in the presence of M-HA and Skinkò E. Both the treatments were effective but Skinkò E reduced NF-kB and HO-1 expression 3,3-fold and 2,6-fold, respectively, compared with M-HA alone (the data are statistically significant).

### 3.4. Oxidative Protein Damage

As further biomarker of the oxidative stress we evaluated the protein expression of the *γ*-H2AX (primary antibody anti-*γ*H2AX: Cat No. 05-636 from Millipore, MA, USA), through western blotting analysis following the procedure described in the previous section. The quantification of carbonyl groups introduced into proteins by oxidative reactions was detected by OxyBlot kit (data not shown). Densitometric analysis of *γ*-H2AX (Supplementary File (available here)) showed that M-HA and Skinkò E reduced the protein expression with respect to oxidative stress induced. In particular, both the treatments were effective, but Skinkò E reduced *γ*-H2AX expression 1,7-fold and 1.3-fold with respect to H_2_O_2_ and UV-A, respectively, compared with M-HA that reduced it 1.5 and 1.1 with respect to both oxidative stresses induced.

### 3.5. TBARS Assay

To assess the antioxidant activity,* in vitro* tests were conducted on M-HA and Skinkò E. Human keratinocytes were treated with oxygen peroxide or exposed to UV-A radiation, and TBARS assay (see Figure 5) showed that the levels of lipid peroxidation dramatically increased in response to both H_2_O_2_ and UV-A exposure, whereas M-HA 0,32% w/v reduced the amount of lipid peroxidation. To better unravel the functionality of the diverse components, Skinkò E was subjected to UF treatment on the 3 kDa membrane and both retentate and permeation were tested separately. Retentate contained over 70% of the total HA present, while permeation clearly contained vitamins and components at low molecular weight and a residual HA that proved randomly able to permeate for about 25-30% of total amount contained in the formulation. This particular behavior is known to occur in linear polyanionic polysaccharides that assume specific enlarged conformations in solution, in order to reduce the repulsion forces in between the dimeric repetitive units. When the cells were exposed, simultaneously, to M-HA, Skinkò E and Skinkò E permeate (3 kDa) in the presence of H_2_O_2_ or U-VA, respectively (see Figures 6(a)-6(b)), the levels of lipid peroxidation were substantially reduced with respect to relative positive control. In particular, Skinkò E and Skinkò E permeation significantly reduced lipid peroxidation 1,3- and 1,5-fold with respect to M-HA alone in HaCaT exposed to UV-A (see Figure 6(b)).

### 3.6. Skinkò E Protection against Oxidative Stress-Induced Apoptosis

To further investigate the protection mechanism of Skinkò E treatments against oxidative stress-induced apoptosis, we used a mouse embryonic stem cell line (ES) [33]. In particular, we used an ES cell line which was extremely sensitive to oxidative stress (G6pdΔ ES cells). G6pdΔ is an engineered ES cell line carrying the deletion of the glucose-6-phosphate-dehydrogenase gene. Indeed, G6PD is essential for the production of high levels of NADPH required for the cell detoxification of reactive-oxygen species [22]. We focused on H_2_O_2_ as the oxidant, WT ES, and G6pdΔ ES cells were treated, respectively, with 100mU/ml or 10mU/ml of glucose oxidase (GOX), an enzyme that produces H_2_O_2_ in the cell culture medium, from glucose and water. As shown in Figure 7, Skinkò E, but not M-HA, reverted the effect of GOX, protecting both WT ES and G6pdΔ ES cells against apoptosis. Since SkinkòE protected both WT and G6PD delta from H_2_O_2_ induced apoptosis, we can speculate that molecules present in the formulation can act as antioxidants, bypassing the function normally performed by NADPH.

*Statistical Analysis*. All the data are represented as the mean ± SD. When there was no variability in the values for a group, a one-sample* t*-test was used to compare the group mean to that value; otherwise a two-sample* t*-test was used to compare group means.* p* < 0.05 was considered significant in each of the comparative analyses.

## 4. Discussion

The present experimental study provided consistent information regarding biochemical changes in cells after* in vitro* oxidative damage. This included the potential protective effects, such as, antioxidant activity, not only of M-HA, but also of a formulation based on M-HA plus minerals, amino acids, and vitamins. Due to its rich formulation, the injectable solution of hyaluronic acid, complemented with these small molecules (Skinkò E), demonstrated its efficacy against oxidative stress, which is considered the main cause of skin aging or photoaging. To our knowledge, oxidative damage in terms of H_2_O_2_* in vitro* treatment [32] and UV-A irradiation [33] also contribute to this detrimental condition. To better evaluate the effect of Skinkò E formulation, with respect to the sole M-HA, HaCaT cells were used as the* in vitro* cellular model. Normally, in the skin, oxidative stress is due to reactive-oxygen species (ROS) that can originate both from exogenous factors (i.e., the environment) and from endogenous factors [34, 35]. Specifically* in vitro* tests were carried out to assess the antioxidant activity on M-HA and Skinkò E. Human keratinocytes were treated with oxygen peroxide or exposed to UV-A radiation, showing an increased lipid peroxidation; the latter was significantly reduced by treating the cells with both M-HA and Skinkò E. Interestingly, the beneficial effect was also found when the HaCaT cells were treated with the Skinkò E UF permeation (3 kDa) that consisted of the low molecular weight fraction (vitamins, antioxidants, amino acids, and minerals) [14] and a small amount of residual HA (0,92 mg/ml). In addition,* in vitro* wound healing experiments showed that Skinkò E was superior to the sole HA of the same MW in promoting wound closure, with a relevant and significant improvement that showed in triplicate experiments to accomplish 70% repair in half the time. Beside the UV-A stress* in vitro* model was here tested as discussed by Almeida [29]. Interestingly, this was also prevented by both M-HA and Skinkò E with a marked improvement for the latter that reduced, at transcriptional level, both SOD-2 and HO-1 and protein level NF-kB and HO-1. Since these biomarkers are relevant in assessing the state of the cells, our aim was to highlight the efficacy of the formulations used against the two different oxidative stress insulting conditions tested in this research work. In this respect, our results relative to the decrease of protein biomarkers of oxidative stress (e.g., SOD-2) could be explained through the hypothesis that antioxidants enzymes are activated late following the oxidative stress UV-A induced. In our opinion, the cells survived to the treatment with H_2_O_2_ produced SOD-2 as protective enzyme. While in presence of hyaluronans, the cells do not need to activate it, because specifically both M-HA and Skinkò E are able to counteract ROS production, thus reducing the overall stress that the cells experience. Our observations were supported by the work of Leccia and collaborators [36]. Specifically, they reported that antioxidant enzymes are activated relatively late after the initial UV damage and hence could be considered as ‘‘late-response” genes and proteins. However, the oxidative protein damage was evaluated supporting a lower detrimental action when cells were exposed to (treated with) M-HA and Skinkò E. In addition, the western blot analyses with *γ*-H2AX further support a lower damage to both H_2_O_2_ and UV-A induced stress when the cells received contemporary the treatments. Specifically Skinkò E was permitted to lower damage [37, 38]. The present study confirmed that the use of the intradermal HA solution with other active ingredients may increase keratinocytes function. In particular, amino acids and vitamins present in the Skinkò E formulation are important nutrients to maintain youthful epidermal appearance. For instance, the vitamin B complex is reported to act as free radical scavengers. Also biotin and inositol, important intracellular messengers, play a key role in the synthesis of the matrix proteins forming the cellular scaffolds/ tissue architecture [36]. In addition, antioxidants properties could be also related to the presence of lipoic acid in the formulation tested. The latter, in fact, has been studied for its benefits to skin as potent natural antioxidant [39]. Specifically, lipoic acid improved clinical characteristics related to photoaging of facial skin [40] and also is able to act as protective agent against UV-B induced damage [41]. In* vitro* studies showed its action as ROS scavenger may be accomplished through the direct suppression of the UVR-induced NF-kB activation in human immortalized keratinocytes [42]. In order to test the ability of Skinkò E and M-HA to prevent apoptosis, G6PD delta ES was chosen as cellular model system since they are extremely sensitive to oxidative stress [26]. We have previously demonstrated that it is a reliable model system to analyze apoptosis. Moreover, all the procedures to analyze oxidative stress-induced apoptosis in ES cells have already been set up and described [33]. Using G6pdΔ ES cells, we showed that Skinkò E is also able to protect cells against oxidative induced apoptosis through the production of NADPH, that is, a central enzyme in cell defense against redox insults. Indeed, in order to reduce H_2_O_2_, both essential enzymes, glutathione reductase and catalase, require NADPH; the first enzyme requires NADPH as a cofactor to reduce GSSG in GSH, and the second to form active tetramers out of a single enzymatically inactive subunit. Looking at the Skinkò E formulation, we observed that the three constitutive amino acids of the tripeptide GSH were present in the mix. We can speculate that the presence of these amino acids could induce* de novo* GSH synthesis, supplying cells with new reducing power essential to counteract the oxidative damage. Amino acids and vitamins are also important ingredients for maintaining a youthful appearance. As reported by Tosti [43], the vitamin B complex is essential in different metabolic functions, also acting as free radical scavengers. In addition, the oxidative stress and more generally, the ROS production are among the recognized mechanisms affecting melanocyte disorders which alter skin pigmentation. In particular, Wan and collaborators [44] reported that melanocytes protect skin cells against UV radiation through melanin biosynthesis. Continuous UV radiation exposes melanocytes to oxidative stress and, in this condition, exposed epidermal cells gradually lose this function, resulting in anomalous pigment production [45].

## 5. Conclusions

The present research work suggests a potential role of the Skinkò E formulation on dermal dark spot treatment, in relation to its activity against oxidative stress. Overall the results of this research work confirmed the effectiveness of Skinkò E and of M-HA on cell repair and regeneration through increased cell proliferation and the migration capacity of keratinocytes. It is well known that increased ROS, altering apoptotic pathways, can foster the development of dermatological diseases and aging. Therefore Skinkò E, which protects cells against ROS-induced apoptosis, can play a role in maintaining healthy youthful skin, preventing or delaying skin aging and eventually the onset of skin diseases.

## Figures and Tables

**Figure 1:** Hydrodynamic characterization by SEC-TDA is reported for (a) Skinkò E UF retentate and (b) M-HA.

**Figure 2:** (a) Representative micrograph pictures of HaCaT scratch assays. (b) Repair area percentage for the control and in the presence of treatments: M-HA and Skinkò E; the curves are averages of three different experiments with standard deviation within 5% of the value. (c) Rate of reparation within 96 hours. Skinkò E and M-HA treatments are statistically significant  ^*∗*^(p<0.05) with respect to CTR, Skinkò E and M-HA treatments are statistically significant  ^*∗∗*^(p<0.01) with respect to CTR, and Skinkò E is statistically significant ^§^(p<0.05) with respect to M-HA treatment.

**Figure 3:** Antioxidant biomarkers (SOD-2 and HO-1) were determined by quantitative real-time PCR on HaCaT UV-A pretreated for 4 minutes and subsequently treated with M-HA 0.32% (w/v) and Skinkò E 0.32% (v/v) for 4 hours. Each column represents the mean and error bars represent the standard deviation (n=3). Test-t was performed to evaluate the significance of M-HA and Skinkò E effects with respect to positive control (UV-A),  ^*∗*^p<0.01.

**Figure 4:** Western blotting analyses showed that M-HA and Skinkò E reduce the inflammatory proteins NF-kB and HO-1. In particular, Skinkò E is more efficient than M-HA on these protein modulations.

**Figure 5:** Effect of M-HA 0.32% (w/v) and Skinkò E 0.32% (v/v) on lipid peroxidation after exposure to oxidative stress induced by 50*µ*M H_2_O_2_ for 30 minutes. M-HA and Skinkò E treatments are statistically significant (^*∗*^p<0.01) comparing with the positive control (H_2_O_2_). Also, Skinkò E is statistically significant (^*∗*^p<0.01) with respect to M-HA treatment.

**Figure 6:** Effect of M-HA 0.32% (w/v), Skinkò E 0.32% (v/v), and permeate (3KDa) Skinkò E on lipid peroxidation after exposure to oxidative stress induced by 50*µ*M H_2_O_2_ (a) or UV-A irradiation (b) on HaCaT cells. “∗” in the histogram indicates significant difference at p<0.01, comparing with the Skinkò E and UF Skinkò E Permeate 3kDa treatment groups with respect to M-HA. Data of the amount of lipid peroxides (% respect to CTR) are reported as follows: Graph (a): H_2_O_2_=570±14, M-HA=128±7.0, Skinkò E=95.5±7.7, UF Skinkò E Permeate 3kDa=109±4.2. Graph (b): UV-A=480±14.0, M-HA=114±7.0, Skinkò E=74±5.6, UF Skinkò E Permeate 3kDa=76±7.0.

**Figure 7:** Protective effect of Skinkò E against oxidative stress-induced apoptosis.

**Table 1:** Primer sequences used for the qRT-PCR.

**Gene**	**Forward Primer**	**Reverse Primer**	**AT PCR**
HPRT	5'-TGACCTTGATTTATTTTGCATACC-3'	5'-CGAGCAAGACGTTCAGTCCT-3'	55°C
SOD-2	5'-CTGGACAAACCTCAGCCCTA-3'	5'-TGATGG CTTCCAGCAACTC-3'	55°C
HO-1	5'- GCAGTCAGGCAGAGGGTGATAGAAG-3'	5'- TGGTCCTTGGTGTCATGGGTCAG -3'	55°C

## Supplementary Materials

Supplementary Materials In order to better analyze oxidative stress, *γ*-H2AX (primary antibody anti-*γ*H2AX: Cat No. 05-636 from Millipore, MA, USA) was evaluated as specific biomarker of DNA damage prompted by oxidative stress, through western blotting analysis following the experimental procedure reported in Materials and Methods.
